# Image Super-Resolution Reconstruction Method for Lung Cancer CT-Scanned Images Based on Neural Network

This article has been retracted.

**DOI:** 10.1155/2022/3543531

**Published:** 2022-07-18

**Authors:** Jianming Xu, Weichun Liu, Yang Qin, Guangrong Xu

**Affiliations:** Provincial Key Laboratory of Informational Service for Rural Area of Southwestern Hunan, Shaoyang University, Shaoyang, 422000 Hunan, China

## Abstract

The super-resolution (SR) reconstruction of a single image is an important image synthesis task especially for medical applications. This paper is studying the application of image segmentation for lung cancer images. This research work is utilizing the power of deep learning for resolution reconstruction for lung cancer-based images. At present, the neural networks utilized for image segmentation and classification are suffering from the loss of information where information passes through one layer to another deep layer. The commonly used loss functions include content-based reconstruction loss and generative confrontation network. The sparse coding single-image super-resolution reconstruction algorithm can easily lead to the phenomenon of incorrect geometric structure in the reconstructed image. In order to solve the problem of excessive smoothness and blurring of the reconstructed image edges caused by the introduction of this self-similarity constraint, a two-layer reconstruction framework based on a smooth layer and a texture layer is proposed for a medical application of lung cancer. This method uses a global nonzero gradient number constrained reconstruction model to reconstruct the smooth layer. The proposed sparse coding method is used to reconstruct high-resolution texture images. Finally, a global and local optimization models are used to further improve the quality of the reconstructed image. An adaptive multiscale remote sensing image super-division reconstruction network is designed. The selective core network and adaptive gating unit are integrated to extract and fuse features to obtain a preliminary reconstruction. Through the proposed dual-drive module, the feature prior drive loss and task drive loss are transmitted to the super-resolution network. The proposed work not only improves the subjective visual effect but the robustness has also been enhanced with more accurate construction of edges. The statistical evaluators are used to test the viability of the proposed scheme.

## 1. Introduction

At present, there is an increasing demand for high-resolution images in various fields such as medicine, security, and entertainment [1]. Medical science is the field where images play very important role in diagnosis of the diseases where images are supplied as inputs and output is achieved in terms of identification of the diseases based on images [2]. For example, doctors attempt to identify diseases through high-resolution CT images; diseases are identified through high-resolution surveillance images where similar images can mislead [3]. It is expected that through high-resolution video, healthcare practitioners can obtain more realistic and detailed visual effects to diagnose the diseases and ailments in a detailed manner [4, 5]. The most direct way to increase the resolution is to increase the hardware resolution of the digital image acquisition system [6]. However, high costs and technical bottlenecks often make this method difficult to achieve, and it is not feasible for healthcare practitioners to devise these computational methods to enhance the quality of the images of patients [7]. Therefore, obtaining high-resolution images under unified hardware conditions is the focus of super-resolution reconstruction technology [8]. Super-resolution reconstruction technology provides an effective way to solve this problem. Spatially modulated full-polarization imaging technology is following the traditional methods to fetch the information from the image [9]. A new system of polarization imaging technology has been evolved from the time-sharing and simultaneous polarization imaging technology [10]. Under the new imaging system, the system uses the Savart polarizer to modulate the four Stokes vectors of the detected target in the same interference image, so as to pass a single image as an input [11].

The complete polarization information can be obtained by acquisition [12]. The system has gradually become a research hotspot due to its advantages of obtaining multiple Stokes vectors at the same time, simple structure, and easy implementation with respect to dynamic targets [13]. A direct mapping function is established between the sensor pixels and the scene to obtain enhanced images with the new computational imaging system [14]. The feature extraction and image reconstruction as a whole is devised using the adaptive and the latest methods. The newer systems can use high-performance computing power and global information processing capabilities to enhance the resolution of the images and to extract the relevant information from the images [15, 16]. It plays a role in applications such as ultra-diffraction-limit imaging, high resolution (HR) imaging with a large field of view, and clear imaging through scattering media [17]. Single-image super-resolution technology uses a single degraded low-resolution image to reconstruct a high-resolution image [18]. High-resolution images have more details, and these details are of great significance in practical applications such as diagnosis of diseases [19]. Image super-resolution technology has always been a research hotspot in aerospace, remote sensing, target recognition, and other fields [20]. Image super-resolution (SR) technology has been widely applied, with high practical value in medical imaging, face recognition, high-definition audio, video, and other fields. Until now, medical imaging has played an important role in the medical field. High-resolution medical images can improve the work efficiency of doctors and reduce the rate of missed diagnosis. CT images are often used in guided radiotherapy, so it is of great significance to obtain high-resolution CT images.

In [2], authors have proposed super-resolution technology for the first time. At present, super-resolution technology is divided into three categories: interpolation-based methods, reconstruction-based methods, and learning-based methods. The learning-based method can introduce more high-frequency information than the other two types of methods and can obtain better robustness to noise. In [3], optical remote sensing image super-resolution reconstruction technology is used that processes one or more low-resolution optical remote sensing images with complementary information to obtain high-resolution optical remote sensing images. Optical remote sensing image is the data support and application basis of remote sensing image target detection, providing rich information for monitoring the images to extract the hidden information. Therefore, it is of great significance to improve the resolution of remote sensing images. Optical remote sensing image reconstruction algorithms are divided into two categories; one is human-centered methods, and the other is machine-centered methods. Human-centered methods often use PSNR (peak signal-to-noise ratio) and SSIM (structural similarity) as evaluation indicators and generate visually satisfactory pictures for recognition. Usually this type of method ignores the follow-up due to the particularity of computer vision tasks (such as target detection and classification). The machine-centric method has many options, and the machine learning-based algorithms enhance the quality of the image for drawing useful information from the images by training the algorithm on huge data set of images.

The newly developed methods take the execution result of the computer vision task as an optimization index and evaluate the reconstruction performance of the algorithm through the input of images and their respective outputs. The super-resolution reconstruction task is regarded as a preprocessing step for processing the images where the resolution of the images is improved before applying any feature extraction algorithms and classification algorithms [21, 22]. The design principle focuses on learning the resolution invariance of a special task to process multiscale targets in a remote sensing image, so as to facilitate higher-level computer vision task processing and analysis. In the early days, most of the models for SR tasks have been implemented based on interpolation methods, and the most representative of them is the model based on sparse representation [14–16]. These types of models assume that any natural image can be sparsely represented by elements in the image dictionary. Then the model can reconstruct the high-resolution images based on the image dictionary. However, this type of method is computationally complex and requires a lot of computing resources, and this type of method does not perform well in restoring the details of the image. With the development of deep learning, deep neural networks have been introduced into the SR task. SR tasks based on neural networks are implemented in a supervised learning manner. From the perspective of neural networks, it is necessary to establish a pixel-level mapping from low-resolution images to high-resolution images [17]. From a statistical point of view, this process can be considered to establish a conditional probability *p*(*y*|*x*), where *x* is the input low-resolution image and *y* is the corresponding high-resolution image. Through training, the neural network can learn to obtain the statistical characteristics of low-resolution images and restore high-resolution images accordingly, that is, generalize from the training data set to the test data set [18–20]. Image super-resolution reconstruction based on deep neural networks can be roughly divided into two research directions. In order to solve the above problems and generate sharper images, this paper designs a stable and effective energy-based counter-assistance loss based on the commonly used VGG reconstruction loss. Super-resolution (SR) image reconstruction is a technique used to recover a high-resolution image using the cumulative information provided by several low-resolution images. Super-resolution reconstruction of sequence remote sensing image is a technology which handles multiple low-resolution images to provide a better quality image irrespective of the underlying hardware. This technology works purely independently without the involvement of hardware support, and once the low-resolution images are enhanced by using this super-resolution technology, the images can be used on any machine; they will be classified in an accurate manner irrespective of the hardware configuration of the machine.

The advantage of using an energy function as a discriminator to replace the traditional discriminator is that the process of encoding data into energy takes into account the volatility of the neural network itself, and after the energy flow of the data is constructed, the generator can be used to track the energy flow. Another advantage of tracking the energy flow of data is that when the energy approaches 0, the discriminator no longer generates additional gradients, so the energy-based confrontation generation network is relatively stable. In order to construct a relatively stable auxiliary energy loss, this article draws on the concept of Boltzmann distribution in statistical mechanics and the energy-based GAN model [19]; the Boltzmann distribution establishes the relationship between energy and probability. According to this distribution, the lower the energy, the greater the probability of the corresponding sample to find a matching image. When the loss function converges, the curve tends to be flat. The corresponding probability distribution can be considered as the distribution Pdata of real data. Therefore, it is assumed that samples that obey the data distribution have low energy. Then when the energy of the sample that passed to the discriminator is low enough, it can be considered that the sample obeys the data distribution and the generated confrontation network can be regarded as the energy flow of tracking the data using the model distribution.

For spatially modulated computational imaging, the image degradation process not only includes the direct mapping model between the sensor pixel and the scene in the traditional imaging method, and the mapping relationship corresponds to the interference fringe intensity image on the CCD of the spatially modulated full-polarization computational imaging; it also includes the use of two-dimensional discrete Fourier transform to transform the spatial domain interference fringe information into the frequency domain computational imaging and the use of low-pass filter calculation to obtain the target's Stokes vector information spatial modulation process [2]. At the same time, in the hyperspectral full polarization imaging system, in addition to obtaining the polarization information of the detection target, it is also very important to obtain the Hyperspectral Information and high-resolution visible panchromatic image of the target. These heterogeneous redundant hyperspectral and visible light images are the low resolution of the same target scene. The polarized image SR method provides additional target scene priors. Interpolation-based methods for super resolutions are also explored by the researchers in the existing literature. These methods use the pixel values of adjacent pixels in the image space domain to determine the pixel values of the points to be interpolated. The most common ones are the nearest neighbor interpolation, bilinear interpolation, and bicubic interpolation. The existing literature proposes spatial nonlinear interpolation algorithms, wavelet-based algorithms, and bilinear interpolation-based methods [10–12] as interpolation-based image super-resolution reconstruction method is easy to process, but due to the lack of sufficient prior knowledge and image observation model, the reconstructed image has blurred edges and poor overall visual effect.

In recent years, transfer learning methods [15, 16] have provided ideas and technical means for using scene priors to perform SR. The representative method is to use HR RGB image prior information to enhance hyperspectral image SR [17–19]. In actual imaging detection, hyperspectral imaging systems often sacrifice time and spatial resolution in order to achieve high spectral resolution, while visible light (or multispectral) cameras integrate radiation with a wide wavelength range, which can easily capture high spatial resolution in real-time images. Inspired by this, this article focuses on the spatial modulation type computational imaging degradation process for lung cancer images. The characteristics of the imaging system are utilized for preparing the model. The convolutional neural networks (CNNs) are utilized with new architecture in the proposed framework where the hybrid mechanism is used by fusion of spatial modulation-based computational imaging method based on scene feature migration.

In order to solve the problem of excessive smoothness and blurring of the reconstructed image edges caused by the introduction of this self-similarity constraint, a two-layer reconstruction framework based on a smooth layer and a texture layer is proposed for a medical application of lung cancer. This method uses a global nonzero gradient number constrained reconstruction model to reconstruct the smooth layer. The proposed sparse coding method is used to reconstruct high-resolution texture images. Finally, a global and local optimization models are used to further improve the quality of the reconstructed image.

The dual-drive adaptive remote sensing image for target detection is based on the characteristics of optical remote sensing images. An adaptive multiscale remote sensing image super-division reconstruction network is designed. The adaptive feature terminology is used as a flexible feature of the proposed approach which works well on all type of low-resolution images by employing super-resolution technology without caring about the hardware and software details. Any images can be supplied as input images, and the adaptive feature technology is able to extract the features from the image to assist in enhancement of its resolution and to assist in classifying the image more accurately. The selective core network and adaptive gating unit are integrated to extract and fuse features to obtain a preliminary reconstruction. Through the proposed dual-drive module, the feature prior drive loss and task drive loss are transmitted to the super-resolution network. Due to the precision of the remote sensing image target detection task, the super-division network can better serve the target detection task and improve the performance of target detection for serious diseases like lung cancer from the available images. The proposed work not only improves the subjective visual effect, but the robustness has also been enhanced with more accurate construction of edges.

## 2. Existing Frameworks

### 2.1. Spatial Modulation Type Hyperspectral Full-Polarization System

Spatial modulation type full-polarization imaging is a new type of polarization imaging systems developed next to the traditional time-sharing and simultaneous polarization imaging systems.  Figure 1 shows a 2-channel hyperspectral full-polarization simultaneous imager. The system is mainly composed of pre-expanded optic devices (beam expander optics (BEO)), half-wave plate front surface aperture diaphragm (S), Savart polariscope (SP), liquid crystal tuning filter (P), computing imaging system (CIS), and CCD. Among them, the area array detector has a resolution of 2048 × 2048 in the visible near infrared band and a pixel size of 12 *μ*m; the short-wave infrared band has a resolution of 640 × 512 and a pixel size of 20 *μ*m.

The imaging system adopts the principle of spatial modulation of Stokes vectors and modulates 4 Stokes vectors (S03~S) in the same image at the same time. One acquisition can obtain modulation information containing the 4 Stokes vectors of the target. Based on this, it can be parsed out. The realization of hyperspectrum can quickly switch the band through the liquid crystal tuning filter and realize the rapid measurement of the complete polarization state of the target which can reflect the scene and target information from different angles.

### 2.2. Image Degradation Model

Let {*g*1, *g*2, ⋯, *gn*} be *n* frames of low-resolution images collected by existing hardware devices, and *f* is the high-resolution image to be reconstructed. As shown in Figure 2, the high-resolution image in Figure 2(a) is transformed into the result in Figure 2(b) after geometric transformation Tk, and then Figures 2(a) and 2(b) are, respectively, blurred (point spread function Hk and downsampling D); add noise to get Figures 2(c) and 2(d). Consistent with literature [11], the image degradation model is expressed as:

(1) $$\begin{array}{c} g_{k}={DH}_{k}T_{k}f+\eta_{k},k=1,2,\cdots ,n. \end{array}$$

In Equation (1), Tk is the geometric transformation, Hk is the point spread function, *D* is the downsampling operator, and *η*k is the noise signal. In this paper, 4 × 4 times reconstruction is considered, so the downsampling operator *D* is 4 : 1 sampling.

In order to obtain a more accurate degradation model, it is necessary to study the corresponding relationship between the high-resolution coordinate system and the low-resolution coordinate system. For this reason, it is specified that the upper left corner of the image is the origin of the coordinate, the right is the positive direction of the *x*-axis, and the downward is the positive direction of the *y*-axis. The positions of the pixels indicated by the dots in Figures 2(a), 2(b), and 2(d) in the corresponding coordinate system are shown in Figures 2(a), 2(b), and 2(d).  Figure 2(d) is the positional relationship of the pixels shown by the dots in Figure 2(d) in the low-resolution coordinate system, and its coordinates are (*s*, *t*); Figure 2(b) is the position of the dots in Figure 2(b) shows the positional relationship of the pixel in the high-resolution coordinate system. Its coordinates are (*x*0, *y*0). After downsampling, (*x*0, *y*0) becomes (*s*, *t*), which is the gray value of (*s*, *t*). It is determined by the blur of the point spread function Hk at (*x*0, *y*0); Figure 2(a) is the positional relationship of the pixel shown by the dot in Figure 1 in the high-resolution coordinate system, and its coordinates are (*x* + *ex*, *y* + *ey*); after the transformation *fk* = *Tkf*, it becomes (*x*0, *y*0); Figure 2(c) is a partial enlarged view of the box part in Figure 2(a), and the errors in the *x* and *y* directions are respectively. In addition, since the point spread function Hk does not change the positional relationship of the coordinates, the process from Figures 2(b)to 2(d)) does not reflect Hk.

Therefore, the accurate degradation process can be described as

(2) $$\begin{array}{c} g_{k}\left(s,t\right)=H_{k}T_{k}f\left(x+e_{x},y+e_{y}\right)+\eta_{k}. \end{array}$$

In Equation (2), (*s*, *t*) = DTk(*x* + *ex*, *y* + *ey*). Here, the gray value at the position (*s*, *t*) in the low-resolution grid is not only determined by the high-resolution grid (*x* + *ex*, *y* + *ey*) but is determined by the position and the surrounding pixels. The determination method depends on the point spread function Hk. Considering that the acquisition process of low-resolution images is the overall acquisition of the same scene; it may be assumed that the transformation Tk is an overall transformation. In addition, assuming that the point spread function Hk has translation invariance, then the resolution is represented by

(3) $$\begin{array}{c} H_{k}T_{k}\left(x^{\prime },y^{\prime }\right)=H_{k}f\left(x+e_{x},y+e_{y}\right). \end{array}$$

Considering that *fk* = *Tkf*, thus forming

(4) $$\begin{array}{c} g_{k}\left(s,t\right)=H_{k}f\left(x+e_{x},y+e_{y}\right)+\eta_{k}. \end{array}$$

Since |*ex*| and |*ey*| will not exceed half a pixel unit, the above model is usually approximated by

(5) $$\begin{array}{c} g_{k}\left(s,t\right)\approx H_{k}f\left(x,y\right)+\eta_{k}. \end{array}$$

Assuming that the point spread function remains unchanged during the image degradation process, and the filter *h* is approximated instead, two image degradation models in the spatial domain can be obtained:

(6) $$\begin{array}{c} g_{k}\left(s,t\right)=h*f\left(x+e_{x},y+e_{y}\right)+\eta_{k}, \end{array}$$

(7) $$\begin{array}{c} g_{k}\left(s,t\right)\approx h*f\left(x,y\right)+\eta_{k}. \end{array}$$

In Equations (6) and (7), “∗” is convolution, (*s*, *t*) = DTk(*x* + *ex*, *y* + *ey*) ≈ DTk(*x*, *y*). Equation (5) retains subpixel information, and Equation (6) is approximated by rounding. Ignore this information. In the process of super-resolution reconstruction, literature [11–14] all use Equation (6) as the image degradation model, directly discarding the subpixel information which will inevitably affect the accuracy of the reconstruction model. This paper tries to base on the degradation model (5) which establishes a super-resolution reconstruction model based on subpixel displacement to improve the accuracy of the reconstruction model.

## 3. Model Building Using the CNN-Based Hybrid Mechanism

### 3.1. Sparse Coding Model

This paper proposes a dual-drive adaptive multiscale super-division reconstruction algorithm for target detection which mainly utilizes an adaptive multiscale super-division reconstruction method for enhancing the image quality of the degraded images of lung cancers. The specific structure is shown in Figure 3. The low-resolution remote sensing (ILR) image first obtains the reconstructed super-division image ISR through the adaptive multiscale method specially designed for remote sensing images. This module contains the adaptive multiscale feature extraction block and integrates the optional multiscale. The feature extraction and feature gating units can flexibly fuse the multiscale features of remote sensing images and enhance the target features. Then the super-division image ISR and the original high-resolution image IHR are sent to the feature-driven prior module for feature alignment, and the feature-driven loss is passed into the super-division reconstruction network to guide the generation of super-divisions that are more suitable for target detection of remote sensing images. Then, considering the particularity of the subsequent target task, send the super-divided optical remote sensing image to the task driving module, that is, the target detection module, and pass the task driving loss to the previous super-dividing network to obtain the final remote sensing images detection result. The overall structure is shown in Figure 4 with lung cancer image of CT scan.

### 3.2. Sparse Coding Unit

Recent studies have shown that the traditional sparse coding considering the geometric structure of the image in sparse coding improves the sparse coding ability [15]. A priori condition for image geometric structure is that the natural images often contain repeated structural blocks. However, due to the potential instability of sparse coding methods, image blocks with similar geometric structures often have different sparse coefficients, resulting in flaws in the reconstruction results which can be eliminated by proposing more potential solutions. Therefore, it is necessary to use the nonlocal self-similarity of the image to stabilize the sparse coding. Rahman et al. [16] have proposed a hypothesis based on nonlocal self-similarity; if in a nonlocal neighborhood, the image block ×*j* is the *j*th of the *k* most similar to the image block ×*j*, then in the same the nonlocal neighborhood corresponding to the sparsity coefficient, Sj is also the *j*th most similar sparsity of Sj. This nonlocal self-similar prior condition is defined:

(8) $$\begin{array}{c} \varepsilon_{1}=\overset{n}{\underset{i=1}{\sum }}{\left\|s_{i}-\underset{j}{\sum }\omega_{ji}s_{j}\right\|}_{2}^{2}={\left\|S-SW\right\|}_{2}^{2}, \end{array}$$

where *ω*_*ji*_ is the self-similar weight of ×*j* relative to ×*j*, in *ω*_*ji*_ = *ω*_*ji*_ = *c*_*i*_ · *e*((‖*x*_*i*_ − *x*_*j*_‖^2^)/(*h*_*i*_)) definition, hj is a smoothing parameter, and cj is a normalized parameter.

(9) $$\begin{array}{c} W_{ji}=\left\{\begin{array}{c} \omega_{ji},\\ 0,otherwise. \end{array}\right. \end{array}$$

If xj belongs to the *k* blocks most similar to xj, combine Equation (8) with the traditional sparse coding model in Equation (9) to obtain a nonlocal self-similar sparse coding model as shown:

(10) $$\begin{array}{c} \arg\underset{D,S}{\min}{\left\|X-DS\right\|}_{F}^{2}+\lambda \overset{n}{\underset{i=1}{\sum }}{\left\|s_{i}\right\|}_{1}+\lambda_{1}{\left\|S-SW\right\|}_{2}^{2}, \end{array}$$

where *s*.*t*.‖*d*_*i*_‖^2^ ≤ *c*, *i* = 1, 2, ⋯*k*.

The sparse coding model pays attention to the sparse coefficient space, uses the self-similarity of sparse coefficients to reduce the error of sparse representation, and protects the geometric structure of the image but does not pay attention to the choice of dictionary training. A good training dictionary can reduce rebuild defects and improve the quality of reconstructed images. The dictionaries obtained by training the sparse coding model of Equations (9) and (10) lack orthogonality and have redundancy which weakens the effectiveness and stability of the dictionary. It also reduces the reconstruction efficiency and reconstruction accuracy and easily leads to the inaccuracy of the reconstructed geometric structure. It is necessary to introduce the noncorrelation constraint of the dictionary to reduce the inaccuracy of the reconstructed geometric structure and improve the quality of the reconstruction result. This nonrelevance constraint is defined as follows:

(11) $$\begin{array}{c} \varepsilon_{2}={\left\|D^{T}D-I\right\|}_{2}^{2}. \end{array}$$

In Equation (11), *I* ∈ *Rk* × *k* is the identity matrix, and *D*^*T*^ is the transposed matrix of dictionary *D*. When any two atoms in the dictionary are orthogonal, *ε*2 = 0, at this time, the noncorrelation of the dictionary is the highest. Introducing Equations (8) and (11) into the traditional sparse coding model, the resulting sparse coding model is shown as

(12) $$\begin{array}{c} \arg\underset{D}{\min}{\left\|X-DS\right\|}_{F}^{2}+\lambda_{2}. \end{array}$$

The solution of Equation (12) is divided into two parts: fixed dictionary *D* to solve the sparse coefficient *S* and fixed sparse coefficient *S* to solve the dictionary *D*. Fixed dictionary *D* solves the sparse coefficient *S*; Equation (12) becomes the following formula as shown.

(13) $$\begin{array}{c} \arg\underset{S}{\min}{\left\|X-DS\right\|}_{F}^{2}+\lambda \overset{n}{\underset{i=1}{\sum }}{\left\|s_{i}\right\|}_{1}+\lambda_{1}{\left\|s-sw\right\|}_{2}^{2}. \end{array}$$

Use feature search algorithm to update sj one by one. The fixed sparse coefficient *S* is used to solve the dictionary *D* with a fixed sparse coefficient *S*, and Equation (13) leads to the following equation:

(14) $$\begin{array}{c} \arg\underset{D}{\min}{\left\|X-DS\right\|}_{F}^{2}+\lambda_{2}{\left\|D^{T}D-I\right\|}_{2}^{2}. \end{array}$$

### 3.3. Adaptive Feature Gating

In order to obtain a better reconstruction effect and reduce calculations, it is necessary to add an adaptive gating unit between the selectable multiscale feature extraction layers to adapt to the complex nonlinear mapping relationship during remote sensing image reconstruction which reduces the redundant information. Therefore, in the process of feature transfer, we adopt a simple adaptive gating mechanism to solve the redundant information in the process of feature transfer and increase the flexibility of the network. The adaptive feature gating unit is shown in Figure 5. The key to adaptive feature gating is to adaptively obtain the gate control score of the input feature map *M*_*i*−1_. When the gate control score (*M*_*i*−1_) is determined, it provides detail on how much feature information needs to be retained. The characteristic information is retained as

(15) $$\begin{array}{c} M_{i-1}^{\prime }=M_{i-1}*Score\left(M_{i-1}\right). \end{array}$$

In order to calculate the gating score, we first use the global average pooling operation to reduce the dimensionality of the feature map and then add two full connections connected to BN as a simple nonlinear mapping function, and a ReLU function is utilized to capture the dependence between channels. Finally after the Softmax operation, the vector *G* containing two elements is output. The element with a larger value is recorded as the gated score of the feature map *M*_*i*−1_.

### 3.4. Dual-Drive Module

We know that the quality of optical remote sensing image target detection results depends largely on the clear image and sufficient texture information to extract specific feature information. Therefore, a dual-drive module (DDM) is proposed, and feature priority drive (FPD) and task drive (TD) are added to reduce the feature gap between super-resolution images and real high-resolution images. We combine the target detection network and the super-division reconstruction network for joint training to make the super-division reconstruction model more suitable for target detection and provide a solution for the remote sensing image super-division reconstruction method for target detection. The dual-drive module consists of two parts, a characteristic a priori-driven part and a task-driven part. In order to reduce the feature gap between the super-resolution image and the real high-resolution image, we first add the feature prior drive and use the trained mask R-CNN with ResNet50-C4 [15] as the feature extractor since mask R-CNN introduces mask reflection and it has no transitional coupling with subsequent detectors which helps to improve the usability of the generated image in other detection networks. After feature alignment, the loss is passed to the previous super-division reconstruction network to constrain the characteristics of the super-division reconstruction image to be as similar as possible to the characteristics of the real image.

Then, it is observed that the feature gap between the super remote sensing image and the real high-resolution image is reduced. The feature prior drive is a result of relying on empirical selection but lacks flexibility and adaptability. Therefore, in order to fully explore the interaction between the super-division network and target detection, we also add task driving to jointly train the target detection network and the adaptive multiscale super-division reconstruction network. Explicitly include the task driving loss Ltask in the training of the adaptive multiscale super-division reconstruction network.

## 4. Experimental Outcome

### 4.1. Comparative Experiment

The comparative study is made in order to evaluate the results of the proposed approach with the existing methods. We have selected several mainstream representative super-division reconstruction methods and magnified the image by 2 times for comparison experiments. The detection performance of these super-reconstructed images is tested on the UCAS-AOD data set, and then in second phase, these are tested on the lung cancer data set taken from the Zhongnan University Xiangya Medical College. The detection networks selected by the comparison method are the same as this method, and all use the Faster R-CNN network with FPN.  Table 1 shows the PSNR values of optical remote sensing images reconstructed by different methods and the results of the detection performance AP (average precision) of these images. APS, APM, and APL represent the detection performance of small, medium, and large-scale targets, respectively.

As shown in Table 1 in case of double downsampling, the AP decreases from 47.6% to 22.14%. It can be seen that the performance of the super-resolution reconstruction network has a great impact on the detection results of the target detection network Faster R-CNN. Small-scale and mesoscale targets are greatly affected. The APS is reduced from 21.5% to 6.71%, and the APM is reduced from 48.5% to 23.46%, respectively. According to the analysis, this is caused by the loss of multiscale information and the limitation of downstream target detection tasks. We have utilized an adaptive multiscale super-division reconstruction module and a dual-driver module to reconstruct the multi-scale information of the image and also to significantly improve the performance of remote sensing image target detection. Our method has an AP value of 44.89% and the original high resolution. The image detection result is only 2.71% which shows the effectiveness of our method. The detection effect of small-scale targets is improved more obviously, and the APS is increased from 6.71% to 20.3%.

It can be seen from Tables 1–2 that both MSRN and AMFFN use multiscale methods to reconstruct super-resolution remote sensing images, but their multiscale networks are fixed which cannot guarantee the extraction of the multi-scale information of optical remote sensing images. The subsequent target detection task is difficult; hence, there are serious shortcomings in both the results of reconstruction effect and the target detection effect. The results are evaluated on two data sets as mentioned in the tabular results. Our method has an average increase of 1.38 dB and 1.67 dB, respectively, in resolution, and mAP increased by 10.67% and 10.3% on an average, respectively, which shows the effectiveness of the adaptive multiscale super-division reconstruction module and the dual-drive module for improving the quality of the images. VDSR uses the loss of the detection network to optimize the previous super-resolution network D-DBPN to improve the performance of target detection, but the deep VDSR network structure may cause problems such as the disappearance of the gradient. FDSR only uses the feature extractor to align the original image features with the reconstructed image features and then transfers the alignment loss to the previous D-DBPN network. This method has great limitations. The detection accuracy of the above two methods is a little higher than that of the conventional super-resolution method. However, the above two methods do not take into account the characteristics of optical remote sensing images, so the reconstruction effect is general. On the above two data sets, the average detection accuracy mAP of these methods is 62.96% and 63.91%, but the PSNR is only 26.62 dB and 26.80 dB. Taking into account the advantages and disadvantages of these two methods, we have introduced dual-drive modules, combined with feature prior drive and task drive. In proposed method, the PSNR reached to 28.75 dB and 28.58 dB on the UCAS-AOD data set and lung cancer data set, respectively. VDSR and FDSR are 2 dB higher on average, and the target detection accuracy mAP is improved more obviously reaching 69.67% and 68.61% which shows that our method has greatly improved the reconstruction effect and detection accuracy.

In order to better verify the superiority of our method, we also selected representative test results on the UCAS-AOD and lung cancer data sets for visual display. In the test result, the red box indicates missed inspection, and the yellow box indicates the wrong test result. It can be seen from the Figure 5 that other methods have error detection and missed detection to varying degrees, and our method has good detection results. In summary, our method has the best overall performance. It not only has a better reconstruction effect on optical remote sensing images with diverse scales, but also has a great improvement in detection accuracy.

### 4.2. Convergence Curve Comparison

In order to verify the effectiveness of the key components of the proposed algorithm model, this section conducts sufficient ablation experiments. The first is to discuss the impact of the number of feedback loops, that is, the number of recursive DCB modules T and the number of MRB modules N in the DCB module on performance and then the impact of global feature fusion (GFF) and multicore fusion module (MKFB) on performance in structural design. It should be noted that in order to speed up the training process and ensure the fairness of the result comparison, all ablation experiments in this section only use the DIV2K data set as the training set, the Set5 data set as the test set, and the magnification factor is 4.

(1) In the analysis of the number of feedback *T* and the number of MRB modules *N*, Figures 6 and 7, respectively, show the PSNR index of the reconstruction result of the proposed algorithm under different *T* or *N* conditions, and the result of the DRCN algorithm is used as the benchmark reference value. It can be observed that the larger *T* and *N*, the better the performance of the algorithms.

## 5. Conclusion

In order to solve the problem of excessive smoothness and blurring of the reconstructed image edges caused by the introduction of self-similarity constraints in medical images, this paper proposes a two-layer reconstruction framework based on a smooth layer and a texture layer for providing smooth CT images of lung cancer for better diagnosis. First, in the smooth layer reconstruction, the proposed global nonzero gradient number constrained reconstruction model is used to sharpen the edge of the images and obtain an ideal smooth layer image. The generative model which takes low-resolution images as input, train on ImageNet as the feature extractor, extracts the features of high-resolution images and then builds content-based images. The energy function is utilized for compensating the confrontation loss in the neural network which makes the model more stable and allows the model to generate clear and sharp high-resolution images. The experimental part of this article verifies the effectiveness of the proposed algorithm. The proposed work has achieved mAP (mean average precision) and PSNR (peak signal-to-noise ratio) better than the existing schemes as shown in the result section. The conversion analysis is also optimal as shown in the result section.. The algorithm proposed in this article is attempting to reduce the noise and enhance the image quality for better diagnosis and it can be experimented with more data sets to prove its viability and versatility.

## Figures and Tables

**Figure 1:** Depicting the basic composition of a full-polarization imager.

**Figure 2:** Correspondence between high- and low-resolution coordinate systems.

**Figure 3:** Correspondence between high- and low-resolution coordinate systems.

**Figure 4:** Overall CNN-based network structure for lung cancer-based CT scan images.

**Figure 5:** Adaptive feature gating structure diagram.

**Figure 6:** Convergence curve comparison diagram of different feedback times *T*.

**Figure 7:** Convergence curve comparison diagram of different MRB module number *N*.

**Table 1:** The experimental results of our method for mAP and PSNR with other methods on NWPU VHR-10 data set.

Method	PSNR	mAP
Bicubic	24.74	47.44
MSRN	26.89	57.78
AMFFN	27	58.2
VDSR	26.7	62.85
FDSR	26.84	63.72
Proposed	28.46	68.49

**Table 2:** The experimental results are shown for mAP (mean average precision) and PSNR (peak signal-to-noise ratio).

Method	PSNR	mAP
Bicubic	25.83	48.73
MSRN	27.43	58.85
AMFFN	27.44	59.11
VDSR	26.31	62.84
FDSR	26.53	63.86
Proposed	28.63	69.55

## Data Availability

The data presented in this work can be accessed through PubMed or corresponding author.

## Abbreviations

PSNR: Peak signal-to-noise ratio
AP: Average precision
mAP: Mean average precision
MSRN: Multiscale residual network
VSDR: Very deep super resolution
FDSR: Fuzzy discriminative sparse representation.
